# Drug Treatment Effect Model Based on MODWT and Hawkes Self-Exciting Point Process

**DOI:** 10.1155/2022/4038290

**Published:** 2022-10-14

**Authors:** Xiaokai Nie, Xin Zhao

**Affiliations:** ^1^School of Automation, Southeast University, Nanjing 210096, China; ^2^Key Laboratory of Measurement and Control of Complex Systems of Engineering, Ministry of Education, Southeast University, Nanjing 210096, China; ^3^Shenzhen Research Institute, Southeast University, Shenzhen 518057, China; ^4^School of Mathematics, Southeast University, Nanjing 211189, China

## Abstract

In precision medicine, especially in the pharmacodynamic area, the lack of an adequate long-term drug effect monitoring model leads to a quite low robustness to the instant drug treatment. Modelling the effect of drug based on the monitoring variables is essential to measure the drug benefit and its side effect preciously. In order to model the complex drug behavior in the context of time series, a sin function is selected to describe the basic trend of heart rate variable that is medically monitored. A Hawkes self-exciting point process model is chosen to describe the effect caused by multiple and sequential drug usage at different time points. The model considers the time lag between the drug given time and the drug effect during the whole drug emission period. A cumulative Gamma distribution is employed to describe the time lag effect. Simulation results demonstrate the established model effectively when describing the baseline trend and the drug effect with low noise levels, where the maximal overlap discrete wavelet transformation is utilized for the information decomposition in the frequency zone. The real data of the variables heart rate and drug liquemin from a medical database is analyzed. Instead of the original time series, scale variable s4 is selected according to the Granger cointegration test. The results show that the model accurately characterizes the cumulative drug effect with the Pearson correlation test value as 0.22, which is more significant for the value under 0.1. In the future, the model can be extended to more complicated scenarios through taking into account multiple monitoring variables and different kinds of drugs.

## 1. Introduction

Pharmacokinetics (PK) and pharmacodynamics (PD) are aimed at building mathematical models to extract scientific basis of modern pharmacotherapy. Specifically, pharmacokinetics describes the drug concentration-time courses in body fluids resulting from the intake of a certain dose of drug, and pharmacodynamics describes the observed effect arising from a certain drug concentration [1]. Between PK and PD, PD is more important for describing the variation of body conditions after drug treatment. Following a drug treatment, the original organ function can be enhanced or suppressed. Thus, determining the accurate dosage of the drug is rather essential in the drug prescription. During the treatment process with a given drug dosage, the body condition may be improved but may also suffer some untoward reaction or adverse reaction, including side effect, toxic reaction, allergy reaction, secondary reaction, residual effect, and teratogenesis. Therefore, drug treatment can be helpful to the patient but might be harmful as well, and monitoring the drug effect by observing the clinically monitored variables plays an important role in understanding the mechanism.

The major objective of PD is to explore how the drug influences the monitored variables including heart rate, cardiac output, and mean arterial pressure. Modelling the drug effect can help improve medical precision by applying more suitable treatment for the patient under a target criteria of the monitored variable. Drug effect modelling is critical to realize the online forecasting of the dynamic status of patient's disease. On the other hand, this can reduce the expenditure of medical resources including human resources like physicians and caregivers, drug usage, and economic cost.

Due to the special property of drug effect, the influence of the drug on patient is complex. The instant usage of drug has a long-term and dynamic effect on the patient. For example, there may exist a time delay for some drug to show the medical effects, which may be half an hour in some special circumstances. The time length taken by the drug effect is different not only among different drugs but also for different intake methods. For epinephrine, the effect of intramuscular injection is approximately maintained between 10 and 30 minutes, while the effect of subcutaneous injection can take as long as around 1 hour. Drug effect may increase rapidly and then decrease slowly afterwards before finally vanishes. Before the drug effect vanishes, more drug dosage may be required to be applied to the patient. Besides, multiple drug usages can cause multiple cumulative effects. Determining the correct drug dosage becomes quite challenging as the monitored variables vary with an unpredictable trend. To give a precise dose under a target value of the monitored variable, the whole past drug usage that is still effective should be taken into consideration, as their influence on the patient's future health condition still affects the current required dosage.

In this work, the influence of drug usage on the monitored variables is specifically analyzed, particularly in terms of the cumulative effect from the past drug usage. The rest of the paper is organized as follows: Section 2 gives the research review of drug effect modelling including the state of the art and our contributions, Section 3 presents the method proposed in this research, Sections 4 and 5 show the analysis and the simulation using the real medical data, and Section 6 presents a conclusion of the results and the viewpoints on the further research. All computations are implemented using the software R [2] of the version 4.0.2, and “waveslim” [3] was used for the wavelet decompositions. The hardware platform is iMac Pro (2017) configured with the processor 3.2 GHz 8-Core Intel Xeon W, the memory 32 GB 2666 MHz DDR4, and the Graphics Radeon Pro VEga 56 8 GB.

## 2. Literature Review

The approaches to establishing the models for characterizing the effect of drug on electrocardiogram (ECG) signals like heart rate can be generally divided into three main groups. The pros and cons of the available approaches are compared in detail in the following. The first group includes the typical statistical methods like linear regression, logit regression, analysis of variance (ANOVA) and basic statistical description methods like box plot. In order to study how the choice of anesthetic agent can greatly influence CSF tracer influx, Hablitz et al. [4] used the linear regression analysis. Linear regression with extensions like Lasso, Ridge, and Elastic-net such penalized linear regression methods are good at explanation of the real application background and are simple to understand. Capel et al. [5] used 1- or 2-way ANOVA to investigate the propensity of hydroxychloroquine to cause bradycardia. ANOVA is effective to compare the drug efficiency difference among two or more comparison experiments. In the research of Sun et al. [6], pairwise network meta-analyze was performed using DerSimonian–Laird random effects model to analysis the impact of GLP-1 receptor agonists on blood pressure, heart rate, and hypertension among patients with type 2 diabetes. Gilbert and Krum [7] analyzed the effects of antihyperglycemic drug therapy on heart failure in diabetes by using the meta analysis as well. The pros and cons of this type of methods include that these methods are rather efficient when the data has simple format including cross section data, and the research purpose is more focused on producing the medical experiment results instead of the method improvement. When the data structure is complicated or the objective is lied on the methodology, more interests are concentrated on the subsequent second or third group of methods.

The second type of drug effect models mainly includes machine learning and deep learning methods such as ensemble decision tree methods (AdaBoost or XGBoost), neural networks (convolutional neural network and long-short term neural network), support vector machine, and Bayesian classifiers [8, 9]. For example, Sherman et al. [10] used machine learning methods to identify drug-cancer cell interaction based on some large in vitro databases. Bresso et al. [11] applied the methods decision trees and inductive logic programming to characterizing each drug's side-effect profiles in terms of drug and target properties. Costabal et al. [12] characterized the effect of 30 drugs on the QT interval using Gaussian process regression, sensitivity analysis, and uncertainty quantification. In the research of Juhola et al. [13], several machine learning methods are compared in the analysis of drug effects on iPSC cardiomyocytes, including decision trees, *K*-nearest neighbor nearest searching, multinomial logistic regression, and least squares support vector machines. Results show that random forests classifier and least-squares support vector machines have better performance than the other methods. Ekins et al. [14] compared the performance of different machine learning methods for end-to-end drug discovery and development including Naïve Bayesian, support vector machines, and more recently concerned deep neural networks. Madhukar et al. [15] proposed a Bayesian approach to the drug target identification using diverse data types. Soft computing techniques [16, 17], which although have not been directly applied to the drug effect modelling, can still be the promising solutions to the problem. The pros and cons of this type of methods include the following aspects. It is pretty impressive that the machine learning methods have high prediction accuracy and many of them have reliable generalization. However, most of the machine learning methods are based on quite complex parametric systems and lack of interpretability of parameter meanings, such that may not be the ideal tools for achieving both high accuracy and good explanation.

The third type of drug effect models mainly includes mathematical models such as Cox hazard model based on ordinary differential equations and partial differential equations. Chatterjee and Ahmad [18] applied the fractional-order differential equation model to analyzing the COVID-19 infection of epithelial cells. Huang et al. [19] gave the hierarchical Bayesian inference for HIV dynamic differential equation models which incorporated multiple treatment factors. Thirumalai et al. [20] proposed the fractional differential equations based method to analyze the combined drug therapy for HIV infection. Leander et al. [21] used the stochastic differential equations to analyze the mixed effects involved in pharmacokinetic data of nicotinic acid. Fuentes-Gari et al. [22] have compared the performance of different differential equations in the leukemia treatment, from which it can be found that stochastic differential mixed effects models are useful tools for identifying incomplete or inaccurate model dynamics. In general, those mathematical models have sound performance in both prediction accuracy and explanation.

The motivation of this research is that although the existing results have achieved good performance in PD, especially on drug effect modelling, they still have some shortcomings unsolved due to the complex background of pharmacodynamic, that is, the instant usage of drug can have long and complicated effect on the patient that is shown with the monitored variables. To illustrate this complicated effect, a stochastic modelling approach called Hawkes point process model is introduced to describe stochastic point process. In this work, a Hawkes point process model [23], namely, the self-exciting point process [24] is proposed to characterize the complex drug effect. The essential property of self-exciting point process is the occurrence of any event increased the probability of further events occurring which is consistent with the behavior of drug on patient. This model origins from the area of earthquake behavior analysis [25] and is recently extended to the fields of finance [26], disease prediction [27], and social media [28], where the model has shown satisfactory performance, but it has not been used for drug effect modelling yet.

The acquired data sets of the input variables in this work are time series that have clearly nonstationary property. They are also stochastic time series involved with random noise. Instead of using the original data in the model, the maximum overlap discrete wavelet transform (MODWT) is applied for the feather extraction [29]. MODWT is a method of decomposing the original time series into scaling and wavelet coefficients on different resolution levels, which can be seen as its smooth information and detail information [30]. In this research, these coefficients are used as the deep information involved in the original information. The method Fourier transform [31] can also decompose similar information but it is not suitable for non-stationary time series [32].

The innovation and contribution points in this research mainly have three aspects. The first one and also the main one is that self-exciting point process is proposed to describe the complex behavior of drug on patient. The second one is that MODWT is applied as the feather extraction method to find deep information involved in the original time series. The third one is that the drug effect model developed in this research can describe the effect of a sequence of drug usage on the monitored variables instead of only one usage. The results can be further developed for assisting precision medicine.

## 3. Method

The data contain two variables, the drug usage variable *d*_*i*_ and the monitored variable *x*_*t*_. *d*_*i*_ denotes the *i*th drug dosage at time *t*_*i*_, and *x*_*t*_ gives the value of the monitored variable at time *t*. The goal is to describe *x*_*t*_ by using *d*_*i*_, that is

(1) $$\begin{array}{c} {\hat{x}}_{t}=f\left(d_{i},g\right), \end{array}$$

where *g* represents the other information included in the prediction of *x*_*t*_. In this paper, we mainly analyze the monitored variable heart rate as it is a typical variable that has similar properties to the other monitored variables. Variable *x*_*t*_ such as the changes of the heart rate mainly contains three components: the original waveform change involved in the heart beat change itself, the trend change resulting from the disease, and the trend change arising from the drug usage. In order to keep track of the trend caused by the drug and disease, the wavelet transform method MODWT is applied before implementing the self-exciting point process.

Since the wavelet basis Haar wavelet is simple to understand and has good modelling performance, it is chosen as the basis for the MODWT. The Haar scaling function is defined as

(2) $$\begin{array}{c} \phi \left(t\right)=\left\{\begin{array}{cc} 1 & t\in \left[0,1\right),\\ 0 & \text{else}. \end{array}\right. \end{array}$$

Using dilation and translation, the scaling function at resolution level *j* and location *k* is

(3) $$\begin{array}{c} \phi_{j,k}\left(t\right)=2^{j/2}\phi \left(2^{j}t-k\right). \end{array}$$

For more details, see Graps [33]. Then, the scale variables *s*_*j*,*k*_ can be given by

(4) $$\begin{array}{c} s_{j,k}=<x_{t},\phi_{j,k}>=\int_{R}x_{t}\phi_{j,k}\left(t\right)dt=2^{j/2}\int_{I_{j,k}}x_{t}dt. \end{array}$$

The Haar mother wavelet function *ψ*(*t*) is defined as

(5) $$\begin{array}{c} \psi \left(t\right)=\left\{\begin{array}{cc} 1 & t\in \left[0,0.5\right),\\ -1 & t\in \left[0.5,1\right),\\ 0 & \text{else}. \end{array}\right. \end{array}$$

And the wavelet function at resolution level *j* and location *k* is *ψ*_*j*,*k*_(*t*) = 2^*j*/2^*ψ*(2^*j*^*t* − *k*). The wavelet coefficients *d*_*j*,*k*_ are defined as *d*_*j*,*k*_ = <*x*(*t*), *ψ*_*j*,*k*_>. The scale variables vector *s*_*j*_ = (*s*_*j*,0_, *s*_*j*,1_, ⋯, *s*_*j*,*t*_) and wavelet coefficient vector *d*_*j*_ = (*d*_*j*,0_, *d*_*j*,1_, ⋯, *d*_*j*,*t*_) become new variables which can be used for classification and regression [34, 35]. We name them as scale variables (or scale information) and detail variables (or detail information) in the following sections. For convenience, *s*_*j*,*t*_ is rewritten as *s*_*t*,*j*_. By applying the Haar wavelet to the data *x*_*t*_, the new data *W*_*t*_ is given by

(6) $$\begin{array}{c} W=\left[\left.\begin{array}{ccc} d_{1,1} & \cdots & d_{1,J}\\ d_{2,1} & \cdots & d_{2,J}\\ \vdots & \ddots & \vdots \\ d_{T,1} & \cdots & d_{T,J} \end{array}\right|\begin{array}{ccc} s_{1,1} & \cdots & s_{1,J}\\ s_{2,1} & \cdots & s_{2,J}\\ \vdots & \ddots & \vdots \\ s_{T,1} & \cdots & s_{T,J} \end{array}\right]. \end{array}$$

So far, the step of feature extraction has been finished by using MODWT with the input variables extracted as *W*. Instead of regarding all the variables in *W* as the target variables, Granger cointegration test is performed to verify how the drug influence the variables. The variable with the highest significance is chosen as the final target variable. In the Granger test, we set

(7) $$\begin{array}{c} x_{t}=\overset{m}{\underset{k=1}{\sum }}\alpha_{i}d_{t-i}+\overset{m}{\underset{k=1}{\sum }}\beta_{i}x_{t-i}+\varepsilon_{t}, \end{array}$$

where *ε*_*t*_ is the random noise that follows the Gaussian distribution. Granger test is based on the *F* test, and the hypothesis is defined as

(8) $$\begin{array}{c} H_{0}:\alpha_{1}=\alpha_{2}=\cdots =\alpha_{m}=0, \end{array}$$

and the corresponding *F* statistic is

(9) $$\begin{array}{c} F=\frac{\left({\text{SSR}}_{r}-{\text{SSR}}_{ur}\right)/m}{{\text{SSR}}_{ur}/\left(n-k\right)}, \end{array}$$

where SSR_*r*_ is the residual sum of squares being restricted, and SSR_*ur*_ is that unrestricted. If *F* > *F*_*α*_(*m*, *n* − *k*), then, the hypothesis *H*_0_ that *d*_*t*_ is not the Granger reason of *x*_*t*_ is rejected.

By applying the Granger cointegration test to all the variables in *W*, the most significant variable can be selected as the final target variable, and we can regard the variable as the original *x*_*t*_ without the rest information *g*. In that case, the trend caused by the drug instead of *x* itself or the trend incurred by the disease can be discarded to some extent. For convenience, we still use the symbol *x* to represent the final target variable.

After getting the final target variable *x*, it can be applied to the Hawkes point process involved with the drug information. In the self-exciting point process, the target variable is a number that can be counted, and in this work, we extend it to a continuous context. As a result, the conditional intensity of *x*_*t*_ during the time interval (*t*_*j*_, *t*_*j*+1_) is given by

(10) $$\begin{array}{c} \lambda_{t}=\underset{t_{j}\leq t\leq t_{j+1}}{E}\left[\left.x_{t}-x_{t_{j}}\right|g_{t}\right], \end{array}$$

where *g*_*t*_ includes the information available up to time *t*. After that, a fairly general self-exciting process can be defined in terms of an intensity of the form

(11) $$\begin{array}{c} \lambda_{t}=\mu_{t}+\underset{t_{i}<t}{\sum }\gamma \left(t-t_{i},d_{i}\right), \end{array}$$

where *t*_*i*_ is the time when the *i*th drug usage occurs. *μ*_*t*_ > 0 provides a base level for the process, and we set it as a sin function for simplicity,

(12) $$\begin{array}{c} \mu_{t}=a_{0}+b_{0}\sin\left(\alpha_{0}t+\beta_{0}\right). \end{array}$$

The function *γ*(*t* − *t*_*i*_, *d*_*i*_) ≥ 0 is defined as the exciting kernel of the process, which can be a Gamma distribution. The kernel provides the contribution to the intensity at time *t* that is made by all the previous drug usage events that occur at previous time *t*_*i*_ < *t*, with the associated drug dosage *d*_*i*_. The meaning of the intensity function is that each event increases the intensity and then decays according to the function *γ* until the next drug usage occurs to push it up again. The chosen kernel function is a sigmoid function and a Gamma distribution function with the form as

(13) $$\begin{array}{c} \gamma \left(t-t_{i},d_{i}\right)=\frac{1}{a_{1}+b_{1}e^{-\kappa_{1}\left(m_{1}+d_{i}\right)}}\left\{a_{2}{\left(t-t_{i}\right)}^{\kappa_{2}-1}e^{-b_{2}\left(t-t_{i}\right)}\frac{b_{2}^{\kappa_{2}}}{\Gamma \left(\kappa_{2}\right)}\right\}, \end{array}$$

where *a*_1_, *a*_2_, *b*_1_, *b*_2_, *m*_1_, *κ*_1_, and *κ*_2_ are all parameters to be determined using the real data. In this kernel function, the sigmoid function is proposed to describe the instant drug effect, which we assume the appropriate drug dosage can bring about the corresponding correct effect while using an extra dosage can make little effect when the drug has been already too much or rare. In that case, the sigmoid function is chosen to make it consistent with the assumptions. The Gamma function can be used to describe the trend of the drug effect from the increasing stage to the decreasing stage slowly. It can also describe the decaying process of the drug effect with the time. In the function of *λ*_*t*_, the cumulative of the *γ*(*t* − *t*_*i*_, *d*_*i*_) describes all the previous drug effect until the current time. In order to calculate the parameters *θ* = {*a*_0_, *b*_0_, *α*_0_, *β*_0_, *a*_1_, *a*_2_, *b*_1_, *b*_2_, *m*_1_, *κ*_1_, *κ*_2_}, the ordinary least squares method (OLS) is used to estimate these parameters. The target function to be minimized can be expressed as

(14) $$\begin{array}{c} L=\overset{T}{\underset{t=1}{\sum }}{\left(x_{t}-{\overset{\wedge }{x}}_{t}\right)}^{2}. \end{array}$$

Since ${\hat{x}}_{t}$ is not easy to be obtained, $\Delta {\hat{x}}_{t}$ is used for the replacement of it. Thus, the target function *L* can be given by

(15) $$\begin{array}{c} L\approx \overset{T}{\underset{t=1}{\sum }}{\left(\Delta x_{t}-\Delta {\overset{\wedge }{x}}_{t}\right)}^{2}. \end{array}$$

Replacing $\Delta {\hat{x}}_{t}$ with *λ*_*t*_ in *L* gives

(16) $$\begin{array}{c} L=\overset{T}{\underset{t=1}{\sum }}{\left\{\Delta x_{t}-\left(\mu_{t}+\underset{t_{i}<t}{\sum }\gamma \left(t-t_{i},d_{i}\right)\right)\right\}}^{2}. \end{array}$$

It follows that

(17) $$\begin{array}{c} L=\overset{T}{\underset{t=1}{\sum }}{\left\{\Delta x_{t}-\left(\mu_{t}+\underset{t_{i}<t}{\sum }\frac{1}{a_{1}+b_{1}e^{-\kappa_{1}d_{i}}}\left(a_{2}{\left(t-t_{i}\right)}^{\kappa_{2}-1}e^{-b_{2}\left(t-t_{i}\right)}\frac{b_{2}^{\kappa_{2}}}{\Gamma \left(\kappa_{2}\right)}\right)\right)\right\}}^{2}. \end{array}$$

Taking the derivative of each parameter in *θ*, for parameter *a*_1_, we have

(18) $$\begin{array}{c} a_{1}:\overset{T}{\underset{t=1}{\sum }}\left\{\Delta x_{t}-{\hat{\mu }}_{t}-\underset{t_{i}<t}{\sum }\gamma \left(t-t_{i},d_{i}\right)\right\}\underset{t_{i}<t}{\sum }\frac{\partial \gamma }{\partial a_{1}}\left(t--t_{i},d_{i}\right)=0. \end{array}$$

Similar results can be obtained for the other parameters in *θ*. It is clear that we cannot get a closed form solution from the derivation as the estimated parameters are mutually dependent with each other. Hence, an optimization method of Broyden–Fletcher–Goldfarb–Shanno (BFGS) is proposed to minimize *L*, which is a quasi-Newton method, also known as the variable scale method. This algorithm improves the weakness of Newton's method from the aspects that BFGS will not be easily affected by the initial value without the cost of computing the exact hessian matrix and its inverse in the process of each step of optimization. The NFGS, namely, the Newton improved BFGS, has the characteristic of fast searching of Newton's method and has an improvement in efficient searching for the global optimal solution.

The measurement of the goodness of fit has the metric using *R*^2^, which ranges from 0 to 1, with 1 as the best fit. *R*^2^ has the form as

(19) $$\begin{array}{c} R^{2}=\frac{\text{SST}‐\text{SSE}}{\text{SST}}, \end{array}$$

where SST is the total sum of squares, and SSE is the residual (error) sum of squares,

(20) $$\begin{array}{c} \text{SST}=\overset{T}{\underset{t=1}{\sum }}{\left(\Delta x_{t}-\Delta {\bar{x}}_{t}\right)}^{2}, \end{array}$$

(21) $$\begin{array}{c} \text{SSE}=\overset{T}{\underset{t=1}{\sum }}{\left(\Delta x_{t}-\Delta {\overset{\wedge }{x}}_{t}\right)}^{2}. \end{array}$$

In addition to the *R*^2^, the Pearson correlation test value is also selected for comparison, which is formulated as

(22) $$\begin{array}{c} \text{corr}=\sqrt{\frac{\text{SST}‐\text{SSE}}{\text{SST}}}=R. \end{array}$$

Some other evaluation criteria to assess the performance of the models include mean absolute error and mean percentage error. They all give the measurement of the model fitness, and *R*^2^ and the correlation test can have similar or better effect in measuring the results as their values are constrained in 0 to 1 or -1 to 1, such that the performance can be compared with the significant level. In conclusion, we develop a method to analysis the influence of drug usage on the monitored variable by using self-exciting point process with the kernel function of Gamma distribution.

## 4. Simulation

In this section, we analyze the performance of the method under different noise levels. Since the drug effect can produce the cumulative effect, as shown in Figure 1, we will also analyze how the drug effect influences the model performance. In this Figure 1, the black line represents the cumulative effect ∑_*t*_*i*_−*t*_*γ*(*t* − *t*_*i*_, *d*_*i*_), and the dashed lines represent the separate drug effect *γ*(*t* − *t*_*i*_, *d*_*i*_) for each *i*.

In order to explore how the parameters influence the model performance, the simulation is performed using different parameter settings. The true parameter and the simulated parameters are shown in Table 1. With the parameter given in Table 1, the *R*^2^ results are shown in Figure 2. It can be seen that some parameters have few influence on the *R*^2^, including *b*_1_, *a*_1_, *a*_2_, *b*_0_, *a*_0_. The parameters that have the apparent influence on the *R*^2^ include *b*_2_, *κ*_2_, *κ*_1_, *m*_1_, *b*_0_, *α*_0_, *β*_0_. From Figure 2, it can be seen that when the values of *b*_2_ and *κ*_2_ keep in a fixed ratio around 10, the *R*^2^ keeps in its good performance. When *κ*_1_ increases from 0 to around its best value 0.3, the *R*^2^ increases, but deceases afterwards when *κ*_1_ continues to grow. For the parameter *m*_1_, *R*^2^ has the similar trend. The model performance is not good when *m*_1_ is below its best value but performs relatively well when *m*_1_ is above its best value. For *b*_0_, *α*_0_ and *β*_0_, as they are in the sin function, *R*^2^ shows some kind of routinely performance.

The level of noise also influences the best fitting ability. That is why MODWT is applied before the model training. For example, as shown in Figure 3, by adding the noise which follows the Gaussian distribution, the monitored variable with noise becomes far away from the one without noise. This gap causes the *R*^2^ to be smaller than it should be. By setting the noise level as 0.1 to 10, we can get the best possible *R*^2^ value by choosing the best parameters, and the results are shown in Figure 4. The *R*^2^ decreases as the noise level increases. When the variance of the noise level is bigger than 4, the *R*^2^ decreases below 0.9. When the noise level is 5, the *R*^2^ decreases below 0.8. This result also shows the best possible *R*^2^ under different noise levels.

## 5. Real Data Analysis

The real data we use in this work is the circulatory failure data Hyland et al. [36]. The original source of the data comes from the Medical Information Mart for Intensive Care- (MIMIC-) III database [37], which provides the critical care data of over 40,000 patients admitted to intensive care units at the Beth Israel Deaconess Medical Center. Importantly, MIMIC-III was deidentified, and patient identifiers were removed according to the Health Insurance Portability and Accountability Act Safe Harbor provision. MIMIC-III has been integral in driving large amounts of research in clinical informatics, epidemiology, and machine learning. The data we use contain 812 observations, with 1-minute gap per observation as the resolution level. There are totally 18 variables in the data including heart rate, MAP, cardiac output, and SpO2.

Instead of using all the variables, the variable heart rate is selected as the monitored variable as it has quite few missing values. The minimum and maximum of the heart rate are 61 and 117, respectively. The average and standard deviation are 77 and 9.17, respectively. The drug data in use is the amount of dosage of drug liquemin with unit 5000 U/ml for per dosage. The dosage in use in this real data is 25. The number of usage is 63 times. Liquemin is used to decrease the clotting ability of the blood and help prevent harmful clots from forming in blood vessels. This medicine is sometimes called a blood thinner, although it does not actually thin the blood. Specifically, it is also used in the treatment of heart attacks and unstable angina. Two time-series phases are selected for the real data analysis which contain only liquemin. The flowchart of the proposed method is shown in Figure 5. As shown in Figure 6, the original heart rate variable is transformed by using MODWT to leave out the noise, and the scaling information is selected by using the Granger cointegration test. After that, the scaling information and the drug information are put into the Hawkes point process model with the *R*^2^ or correlation test as the results. In this case, scale variable s4 on resolution level is selected as the target variable *x* according to the Granger cointegration test, and the results are shown in Figure 7. The computed parameters are *θ* = (75, 1.21, 0.13, 1.39, 0.30, 2.08, 0.80, 0.47, 0.0022, 2.77, 0.12). The *R*^2^ is not big as there are other trend inside the original data, but the correlation is obvious with a Pearson test value as 0.22.

Instead of comparing to the time series of the original data, the scale variables on level 4 is compared with the model output since it leaves out most of the noise and with only the trend left for comparison. From Figure 7, we can see that most of the increases and drops are caught by the red line, which means the proposed Hawkes model can effectively measure the drug effect. The Pearson test result is 0.22 that is significantly below the level of 0.1. The obtained model is given by

(23) $$\begin{array}{c} \lambda_{t}=75+1.21\sin\left(0.13t+1.39\right)+\underset{t_{i}<t}{\sum }\frac{1}{0.3+2.08e^{-0.8\left(-0.47+d_{i}\right)}}\left\{0.0022{\left(t-t_{i}\right)}^{1.77}e^{-0.12\left(t-t_{i}\right)}\frac{0.12^{2.77}}{\Gamma \left(2.77\right)}\right\}. \end{array}$$

To sum up, due to the complex development of the monitored variables, there are still some trends caused by the disease that cannot be fully described by our model. We propose a model that gives a different and efficient method for the drug effect measurement in pharmacodynamic.

## 6. Conclusion

In this research, we develop a Hawkes model by using self-exciting point process and sin function to describe the development of medical monitored variable heart rate. Self-exciting point process can describe the effect of the drug and the dosage of the drug. The sin function can describe the basic trend of heart rate. By combining these two functions together, some of the heart rate trend can be described. The model can be used for drug effect prediction and solve the problem of drug precision suggestion. It can also be used for the medical assistant by giving more precise drug dosage description. Specifically, the results show that the model can have a correlation Pearson test to be significant under the significant level of 0.1. The increases and decreases of the trained drug effect can fit the trend of the real drug effect.

The limitations of this research are summarized as the following. In our research, only one kind of drug is modelled, but if many kinds of drug are considered in the model, the model can also be complex. Specifically, in the further research, more complex model can be developed to describe the details of the monitored variable trend including the trend caused by the disease, in addition to the basic trend and drug effect trend. The trend caused by the disease is quite complex to be described but still can be modelled. The analysis of multiple drugs is not simply based on the adding of single drugs, in that case, using many self-exciting point process cannot meet the demand of multiple drug effect analysis. Mutual-exciting point process Hawkes model can be considered to describe the effect of multiple kinds of drug and cumulative drug effect dosage. If multiple drug effect can be modelled, then the further analysis can be concentrated on the inverse problem of drug dosage decision under a predefined monitored variable value.

The proposed modelling solution can be further extended to some other areas in addition to the medical area. For example, in the financial area, the model can be used to monitor the effect of economic events or political events to predict the stock price and security price trend after the event occurs. In the environmental area, the model can be used to monitor the effect of air pollution by decomposing the original time series into three aspects, namely, the basic routine trend, the trend arising from events, and that caused by solar circles. In conclusion, the model developed in this research is an efficient and generalized model for time series data which contains multiple kinds of trends either embraced by the time series itself or caused by the external events.

## Figures and Tables

**Figure 1:** The drug effect of each drug entry. The black solid line represents the cumulative effect, and the dashed lines represent each drug entry.

**Figure 2:** The *R*^2^ under different parameter settings. The true values are shown in Table 1.

**Figure 3:** The simulated monitored variable with noise and the one without noise.

**Figure 4:** The best possible *R*^2^ under different noise levels.

**Figure 5:** The flowchart of the proposed method.

**Figure 6:** The scale variables of the original heart rate time series with drug labelled as the vehicle lines.

**Figure 7:** The scale variables of the original heart rate time series with drug labelled as the vehicle lines.

**Table 1:** Parameter setting under different value.

Parameter	True parameter value	Parameter value range
*a*_0_	70	[1, 100]
*b*_0_	5	[0.1 10]
*α*_0_	1	[0.1 10]
*β*_0_	2	[0.1 10]
*a*_1_	1	[0.1, 50]
*b*_1_	1	[0.01, 10]
*κ*_1_	0.3	[0.01, 1]
*m*_1_	-20	[-100, 98]
*a*_2_	3	[0.01, 10]
*κ*_2_	5	[2.1, 22]
*b*_2_	0.4	[0.01, 2]

## Data Availability

The source code in the method are available from the corresponding author upon request. The real data in application can be requested from Hyland et al. [36].

## Abbreviations

MODWT: Maximal overlap discrete wavelet transform
PK: Pharmacokinetic
PD: Pharmacodynamic
ECG: Electrocardiogram
ANOVA: Analysis of variance
BFGS: Broyden–Fletcher–Goldfarb–Shanno
MIMIC: Medical Information Mart for Intensive Care.
